# Efficacy and Mechanisms of Oleuropein in Postmenopausal Osteoporosis

**DOI:** 10.1155/2022/9767113

**Published:** 2022-08-25

**Authors:** Huilan Liu, Aiguo Zhao, Yulu Huang, Anli Hou, Wenbin Miao, Lu Hong, Nina Deng, Yujuan Fan

**Affiliations:** ^1^Jinan University, China; ^2^Department of Gynaecology, University of Chinese Academy of Sciences Shenzhen Hospital, Shenzhen 518106, China; ^3^Department of Medical Administration, University of Chinese Academy of Sciences Shenzhen Hospital, Shenzhen 518106, China; ^4^Department of Gynaecology, Wuzhou Red Cross Hospital, Wuzhou 543002, China

## Abstract

**Background:**

Postmenopausal osteoporosis (PMOP) has a supernal morbidity rate in elderly females.

**Objective:**

To appraise the effects of oleuropein on bone densitometry, bone metabolic index, oxidative stress, and inflammatory index in PMOP. In addition, the mechanism of olive bittersweet preventing bone loss was explored.

**Methods:**

We grouped 80 salubrious female Sprague-Dawley rats into four teams: (1) sham operation team (sham, *N* = 20), (2) ovariectomy (OVX, *N* = 20), (3) castrated mice fed with oleuropein (OVX+ole, *N* = 20), and (4) castrated mice fed with estrogen (OVX+E2, *N* = 20). The ovariectomized SD rats were continuously raised with 200 *μ*g/kg/dose of oleuropein. Bone mineral density and bone metabolism indexes were recorded. In order to assess the effectiveness of oleuropein on osteopenia, an enzyme-linked immunosorbent assay (ELISA) was devoted to examining the bone marrow indexes. The bone metabolism standards of PMOP rats were appraised by assessing serum levels of calcium, alkaline phosphatase (ALP), phosphorus, malondialdehyde (MDA), and nitrate content by experimental detection methods and levels of osteoclastogenesis inhibitory factor (OPG) and receptor activator for nuclear factor-*κ*B ligand (RANKL) by ELISA. The OPG-RANK-RANKL signal passage was examined by Western blot (WB). We measured bone mineral density using dual-energy X-rays.

**Results:**

Our animal experimental results indicated that oleuropein could significantly improve the bone mineral density of ovariectomized SD rats. In the meantime, it could reduce ending interleukin-6 (IL-6), malondialdehyde (MDA), nitrate, alkaline phosphatase (ALP), and phosphorus (P) serum concentration and would not affect Ca^2+^ concentration. In cell experiments, oleuropein also can promote the proliferation of osteoblasts. Furthermore, it can promote the expression of OPG protein and mRNA. In reverse, it inhibits the expression of RANKL protein and mRNA.

**Conclusion:**

Oleuropein can not only improve the inflammatory and oxidative indexes of castrated rats but also prevent osteoporosis. Oleuropein avoids bone resorption by regulating OPG/RANKL expression.

## 1. Introduction

Postmenopausal osteoporosis (PMOP) is a systemic disease in women, which is mainly manifested as the loss of bone mass and increased risk of bone mass caused by the significant decline of estrogen in the clinic [1]. According to relevant data, more than 200 million women worldwide have osteoporosis. At the same time, the number of fracture patients caused by osteoporosis will double by 2050, which will impose a huge medical and economic burden on the global health system [2]. Currently, estradiol and bisphosphonates are the main methods to prevent PMOP in most hospitals. However, the literature showed that antiosteoporosis drugs have decreased in recent years, especially bisphosphonates [3], because it was highly probable that the drug would increase the incidence of cancer and the risk of osteonecrosis in the patient over the long term [4]. In addition, postmenopausal women could use raloxifene and hormone replacement therapy to prevent osteoporosis [5]. Therefore, due to various side effects of the drug, most postmenopausal women look for natural plant drugs to replace traditional drug therapy.

Components extracted from natural plants are an important origin of new drugs for treating multiple human diseases, including PMOP. Many researchers have demonstrated that the prevalence of carcinoma, coronary artery disease, and osteoporosis [6] is prominently low in the Mediterranean basin [7–9]. People like to eat olive oil on Mediterranean coastal. However, the main component of olive oil is oleuropein, which has been extensively utilized in clinical medicine to resist inflammation, antioxidation [10], and anticarcinogenic effects [11]. Postmenopausal osteoporosis can be alleviated by anti-inflammatory and antioxidant therapy. The Mediterranean diet mainly includes the consumption of olive oil, which includes hydroxytyrosol and oleuropein. The researcher's former experiment displayed that olive oil can delay bone loss, but its functional components are not clear [12].

In this experiment, we fed ovariectomized SD rats with oleuropein to research the resist inflammation, antioxidant, and antiosteoporosis effects of oleuropein. In addition, we also concluded that oleuropein could prevent osteoporosis by regulating the OPG/RANK/RANKL signalling pathway. The results provided a theoretical basis for the effect of oleuropein on preventing osteoporosis and help oleuropein to be widely used in clinical practice in the future.

## 2. Methods and Materials

### 2.1. Medical Ethics

The Medical Ethics Committee approved all animal and cell experimental protocols of the University of Chinese Academy of Sciences Shenzhen Hospital. All SD rats were anesthetized by intraperitoneal injection of 5.2% ketamine for surgery. Animals were managed and raised according to methods provided by the Institutional Animal Care and Use Committee (IACUC).

### 2.2. Animal Experiment Modelling Approach and Treatments

Eighty healthy Specific Pathogen Free (SPF) female Sprague-Dawley (SD) rats were 3 months old. All experimental SD rats were raised at the University of Chinese Academy of Sciences Shenzhen Hospital in ventilated, dry, fixed lighting, and quiet environment. Experimental SD rats were reared in a room with an environmental temperature of 18°C-25°C and humidity of 50%-60%, and they were allowed to eat water freely. After a week of acclimation, 80 SD rats were divided into the sham operation group (20 cases) and the castration group (60 cases). The SD rats were intraperitoneally annotated with 5.2% amiodarone. After the onset of anesthesia, the Y-shaped uterus was found by vertically cutting the middle of the lower abdomen with a scalpel and entering the abdominal cavity. After the bilateral ovaries were found in the abdominal cavity, which was removed, the wound surface of the incision was sutured for hemostasis. Sham surgery was performed to remove bilateral perioophorectomy adipose tissue of the same size as the ovary.

### 2.3. Grouping and Processing of Experimental SD Rats

We grouped 80 salubrious female Sprague-Dawley rats into four teams: (1) sham operation team (sham, *N* = 20), (2) ovariectomy (OVX, *N* = 20), (3) castrated mice fed with oleuropein (OVX+ole, *N* = 20), and (4) castrated mice fed with estrogen (OVX+E2, *N* = 20). The ovariectomized SD rats were continuously raised with 200 *μ*g/kg/dose of oleuropein or 25 *μ*g/kg of estrogen. All experimental SD rats were fed consecutively for 12 weeks according to subgroups.

## 3. Measurement

### 3.1. Bone Metabolism Index in Serum

The blood of the left ventricle of the experimental SD rats was measured, which was centrifuged at 4°C and 2500 rpm for 10 minutes. After centrifugation, the supernatant was placed in Eppendorf tubes and kept at -20°C. The serum should be cooled to room temperature when the automatic biochemical indicator detector was used to detect serum indicators. The serum levels of calcium, phosphorus, malondialdehyde (MDA), and alkaline phosphatase (ALP) were measured by traditional experimental methods. Serum IL-6 values were measured using the ELISA method following the steps of the kit. The contents of osteoclastogenesis inhibitory factor (OPG) and receptor activator for nuclear factor-*κ*B ligand (RANKL) in serum of the four groups were detected by ELISA. The specific operation steps follow the instructions of each kit.

### 3.2. Bone Mineral Density

Measurement of the lumbar spine and left femur bone mineral density (BMD) in SD rats uses dual-energy X-ray (Hologic, Bedford, MA, USA) (S/N806409).

### 3.3. Isolation, Culture, and Passage of Osteoblasts

Three newborn SD suckling rats were taken from the same litter for 48 h to clean the body surface and sacrificed with cervical dislocation. The cranial bone was removed and cleaned with PBS balance solution (at least 3 times) to remove the periosteum, blood vessels, and other connective tissues until the skull became bright and white. The cranial bones were placed in a sterile beaker containing low sugar DMEM and cut into 1 mm × 1 mm pieces with sterile scissors. Add 1 mg/ml of type 2 collagenase into the beaker and digest it for 2 hours at 37°C for 3 times. After digestion, it forms a cell suspension. The cell suspension was centrifuged at 1000 r/min for 10 min, and the supernatant was sucked with a pipette. The precipitated cell clumps were cultured in a culture medium at 5% CO_2_ and 37°C. After the monolayer of cells was covered with a culture flask, digestion was performed with 1 ml 0.25% trypsin, and digestion was terminated with a 10% FBS culture medium. Vials were divided and subcultured, and cells of the third generation were taken for the experiment (Figure 1(a)).

### 3.4. Identification of Osteoblasts

After discarded culture medium was washed with PBS, osteoblasts were fixed with 2.5% glutaraldehyde at room temperature for 10 min. Alkaline phosphatase staining was performed with the NBT/BCIP kit after PBS washing. The morphology, nucleus, and cytoplasm of osteoblasts were observed under an inverted phase contrast microscope (Figure 1(b)).

### 3.5. Drugs Treat Osteoblasts

The osteoblasts were cultured for an alternative time (24 h, 48 h, and 72 h), and the concentrations of 50, 100, 200, and 400 *μ*g/ml oleuropein were added, respectively. The OD value of osteoblasts was detected by the MTT method, and the optimal oleuropein solubility and action time were obtained. The osteoblasts were separated into the blank group (A) and oleuropein group (B) for 48 h culture. The effects of oleuropein on protein and mRNA expression of OPG and RANKL in the compound culture system were measured in groups A and B. The specific operation steps follow the instructions of each kit.

### 3.6. Data Analysis

SPSS 23.0 was used for statistical analysis, and GraphPad Prism 7 (GraphPad Software, CA, USA) was used to visualize the data into required figures. All data were expressed as the mean ± standard deviation (SD). Comparisons between groups were made using an analysis of variance or the LSD method for statistical differences. The comparison between the two groups in accordance with the normal distribution was examined by the *t*-test. The use of *P* < 0.05 stands for statistical difference.

## 4. Results

### 4.1. Changes in Serum Metabolic Indexes and Bone Mineral Density in Experimental SD Rat Ca^2+^ and P

We examined the Ca^2+^ of 4 different groups of mice. We found that the discrepancy had no statistical meaning in Ca^2+^. That implied that Ca^2+^ values in each group did no significant changes (Figure 2(a)). Completely contradictory, compared to the sham group, the P level significantly declined in the OVX+ole group, the OVX group, and OVX+E2 (*P* < 0.05, Figure 2(b)). However, there was no statistical difference in the three groups (*P* > 0.05, Figure 2(b)).

### 4.2. ALP and IL-6

Compared with the other three groups, In the OVX group, the serum interleukin-6 (IL-6) and ALP levels of SD rats were significantly increased (*P* < 0.05, Figures 2(c) and 2(d)). The OVX+ole group and the OVX+E2 group indicated no marked differences between the two indexes, which showed that oleuropein and estrogen probably had the same impact on osteogenesis (*P* > 0.05, Figures 2(c) and 2(d)).

### 4.3. MDA and Nitrate

In the OVX group, MDA and nitrate levels ascended notably. However, in the OVX+ole group, MDA decreased slightly (*P* < 0.05, Figure 2(e)), and nitrate notably decreased. These results exhibited that oleuropein possibly significantly influences antioxidation to avoid bone absorption (*P* < 0.05, Figure 2(f)).

### 4.4. Change of Bone Mineral Density in Experimental SD Rats aft Three Months

The mean bone mineral density of the lumbar vertebra and left femur in the OVX group was lower than that in the other three groups, and the difference was marked dissimilarity (*P* < 0.05). Compared with the OVX+E2 and sham groups, the bone mineral density of the OVX+ole group was no different. It demonstrated that oleuropein had a good effect on maintaining bone mineral density (Figures 3(a) and 3(b)).

### 4.5. Serum OPG/RANKL Indexes

Compared with the other three groups, the serum OPG level in the OVX group was lower (*P* < 0.05, Table 1). Compared with the sham group, OPG levels in the OVX+ole and OVX+E2 groups were decreased, and the differences were statistically significant (*P* < 0.05, Table 1); nevertheless, OPG levels in the latter two groups were not different (*P* > 0.05, Table 1). In contrast with the OVX group, serum RANKL of the sham, OVX+E2, and OVX+ole groups decreased significantly, and the differences were statistically significant (*P* < 0.05, Table 1). In relation to the OVX+E2 group, the RANKL level was lower in the OVX+ole group (*P* < 0.05, Table 1).

### 4.6. Effects of Oleuropein on Osteoblast Proliferation at Different Time Points and Concentrations

Compared with the blank control group, 50, 100, 200, and 400 *μ*g/ml oleuropein had a proliferation effect on osteoblasts, and the dissimilarity was memorably important (*P* < 0.05, Figure 1(c)). After 48 h of treatment, 200 *μ*g/ml oleuropein had the strongest proliferation effect on osteoblasts (*P* < 0.05, Figures 1(a)–1(c)). There was no distinguished distinction in the OD value of osteoblasts after 72 h treatment (*P* > 0.05, Figures 1(a)–1(c)).

### 4.7. Effects of Oleuropein on Protein and mRNA Expression of OPG and RANKL in Osteoblasts

After 200 *μ*l/ml oleuropein was used to culture osteoblasts for 48 h, compared with the blank control group, the expression of OPG protein and mRNA was significantly increased in the experimental group (*P* < 0.05, Figures 4(a) and 4(c)), while the expression of RANKL protein and mRNA was significantly decreased (*P* < 0.05, Figures 4(a) and 4(c)).

## 5. Discussion

The regulation and balance of hormone levels are very important for women's health. An estrogen level that changes dramatically throughout life determines the development of women's age-associated diseases. The hormonal imbalance and estrogen deficiency, resulting in obesity, autoimmune disease, and osteoporosis, greatly increased the risk of fractures during the perimenopausal period. Osteoporosis is a systematic bone disease featured by osteopenia and degeneration of bone microarchitecture, which easily leads to the occurrence of bone fragility and increases the risk of fracture [13]. Osteoporosis and its complications place a huge economic burden on society and, at the same time, pose an unprecedented challenge to the health system as the majority of patients with osteoporosis go untreated [14]. In addition, since the numb of drug treatments for osteoporosis has decreased as a side effect of drugs for osteoporosis, many women are looking for natural plant drugs as alternative therapy [1]. Olive oil is an important part of the Mediterranean diet, which is known for its protective effects on human health. Oleuropein, the most common phenolic compound in olive oil, has a good therapeutic effect on humans' multifarious diseases [15–17]. The result has been clarified in a lot of shown mechanisms and has indicated promising consequences in animal and human studies, especially in PMOP, breast carcinoma, oophoroma, and other disorders [18–20]. Oleuropein is a phenolic compound extracted from natural olive oil, which belongs to iridoids. Currently, there are few studies on the use of oleuropein to prevent postmenopausal osteoporosis.

Our experiment results on animals suggested that oleuropein could significantly avoid BMD descent of ovariectomized SD rats. Besides, it could reduce the levels of serum IL-6, MDA, nitrate, ALP, and P but does not affect the level of Ca^2+^. In osteoblast experiments, oleuropein also can promote the proliferation of osteoblasts. At the same time, it can promote the expression of OPG protein and mRNA. On the contrary, it inhibits the expression of RANKL protein and mRNA.

Ca^2+^ and P are essential elements of the skeleton. 99% of calcium is stored in bone tissue in the form of hydroxyapatite crystals, and 1% of calcium is distributed in body fluids and soft tissues, which are in a dynamic balance [21, 22]. Phosphorus is also an essential element of the human body. 86% of phosphorus is stored in bone tissues in the form of calcium phosphate, and 14% of phosphorus is distributed in important parts of bones and other tissues, which can avoid bone loss and reduce the danger of bone fractures [23]. A lot of studies have also confirmed the important position of calcium and phosphorus in the prevention and treatment of osteoporosis. This study showed that serum phosphorus levels in the OVX group and sham operation group were significantly different (*P* < 0.05). There was no notable dissimilarity in serum phosphorus levels between the OVX group and the OVX+oleuropein group (*P* > 0.05). There was no significant difference in serum calcium levels between the two groups (*P* > 0.05). These results are inconsistent with Saleh and Saleh's research [24], The data showed that the serum P level of SD rats was significantly reduced after OVX, but the serum phosphorus level of OVX rats was not significantly changed after the application of oleuropein. A research study confirmed our view [24]. There were no significant changes in serum calcium levels after OVX in SD rats or in serum calcium solubility after OVX in OVX rats. We consider that such results may be related to the fluctuation of blood calcium content over time during the development of osteoporosis [25].

Stable proliferation between osteoblasts and osteoclasts maintains stable bone metabolism. Osteoblast mineralization plays an essential part in osteoporosis formation of osteoporosis, and ALP activity is very important in the bone formation of osteoblasts because ALP promotes the formation of mineralization matrix proteins of osteoblasts through the hydrolysis of pyrophosphate and inorganic phosphate [26, 27]. This study showed that there were significant differences in serum ALP levels between the OVX group and the OVX+oleuropein group. With significance (*P* < 0.05), the use of oleuropein can significantly reduce the serum ALP level of ovariectomized SD rats. We hypothesized that oleuropein might inhibit mineralization matrix protein formation in osteoblasts by decreasing ALP levels. This mechanism needs further study in our later experiments.

Oxidative stress is also significant pathogenesis of postmenopausal osteoporosis. Reactive oxygen species, for example, MDA, are produced during cell metabolism [28]. Hence, the detected amount of MDA can often reflect the degree of lipid peroxidation in vivo and cell injury. Its level also indirectly reflects the severity of the free radical attack on body cells [29]. The occurrence and development of osteoporosis are often accompanied by oxidative stress and osteoblast apoptosis, whose mechanism is to increase the activity of osteoclasts and promote the apoptosis of osteoblasts and the degradation of bone organic matter [1]. The results of this experiment showed that the serum MDA level of the OVX group had a statistically significant increase (*P* < 0.05). While in the OVX+oleuropein group, the serum MDA level significantly declined. We speculated that oleuropein might reduce the degree of lipid oxidation in vivo by reducing the serum MDA content of ovariectomized SD rats, thereby indirectly reducing the apoptosis of osteoblasts and the degradation of bone organic matter and thus achieving the effect of preventing and treating osteoporosis. Oleuropein had been reported that the viability and dissolvability of nitrate in the blood plasma of ovariectomized rats declined notably after receiving oleuropein [30]. The experimental data showed that the serum nitrate level was significantly reduced after oleuropein treatment (*P* < 0.05). The conclusions reached in this study were consistent with those reported above, but there were no relevant reports explaining the reason, so this result needs to be further explored in our later experiments. Our research results are consistent with the report, but the reason is unclear, and further research is needed.

Our experiment showed that the level of IL-6 in the OVX group was significantly higher than in other groups. The secretion of lymphocytes is the main source of IL-6. Transgenic rats with interleukin-6 overexpression have bone loss and increased bone absorption [31]. Recently, according to relevant literature, IL-6 promotes bone resorption by inducing the proliferation of osteoclasts along the RANKL/RANK/OPG axis [32]. IL-6 can raise the expression of RANKL in osteoblasts [33]. The literature indicated that oleuropein in olive oil could prevent osteoporosis by inhibiting the expression of IL-6 in osteoblasts and decreasing the expression of RANKL in osteoblasts [34, 35]. This view is consistent with the results of this experiment.

The OPG-RANKL-RANK signal system plays an important role in bone remodelling. The proliferation and differentiation mechanism of osteoblasts are affected by the OPG-RANKL-RANK signalling system [36]. Research has shown that anti-RANKL therapy can improve the mechanical properties of bones [37]. High-affinity binding of OPG to RANK acts as an inhibitor of RANK activation, which blocks osteoclast differentiation and inhibits osteoclast function, thereby preventing bone resorption. Therefore, the OPG/RANKL ratio is a lever that modulates the balance between bone resorption and osteogenesis. In postmenopausal women, sudden descent in estrogen secretion results in improved RANKL secretion, declined OPG synthesis, and increased osteoclasts, leading to increased bone resorption and dynamic imbalance of bone remodelling [1]. Data from our animal and cellular experiments indicated that oleuropein could upregulate OPG expression and downregulate RANKL expression, preventing and treating bone loss. At the same time, oleuropein also promoted the proliferation of osteoblasts in a time-dependent manner. Moreover, it is necessary to study a large number of experiments, and there will be more convincing results in the future.

## 6. Conclusion

Oleuropein can not only improve the inflammatory and oxidative indexes of castrated rats but also prevent osteoporosis. Oleuropein avoids bone resorption by regulating OPG/RANKL expression.

## Figures and Tables

**Figure 1:** (a) The third generation of osteoblasts. (b) Osteoblasts stained with alkaline phosphatase. (c) Effects of oleuropein on osteoblast proliferation at different time points and concentrations. After 48 h, the concentration of 200 *μ*g/ml of oleuropein had the strongest effect on osteoblast proliferation (^∗^*P* < 0.05 vs. blank control group (c)).

**Figure 2:** Serum metabolite indexes of different groups at 12 weeks postoperation: (a) comparison of Ca^2+^ level; (b) comparison of P level; (c) comparison of ALP level; (d) comparison of IL-6 level; (e) comparison of MDA level; (f) comparison of nitrate level. Data express the means ± SD (*n* = 20) (^∗^*P* < 0.05,  ^∗∗^*P* < 0.05,  ^∗∗∗^*P* < 0.05 vs. OVX group).

**Figure 3:** Change of BMD in experimental SD rats after three months. (a) Bone density of the lumbar spine. (b) Bone density of left femur. Data represent the means ± standard deviation (SD) (*n* = 20) (^∗^*P* < 0.05,  ^∗∗^*P* < 0.05,  ^∗∗∗^*P* < 0.5 vs. OVX group).

**Figure 4:** (a) Effects of oleuropein on the expression of OPG and RANKL proteins in osteoblasts; (b) representative figure of OPG and RANKL proteins; (c) effects of oleuropein on the expression of OPG and RANKL mRNA in osteoblasts. (^∗^*P* < 0.05 ,^∗∗^*P* < 0.05 vs. blank control group).

**Table 1:** Comparison of OPG/RANKL levels in four groups (mean ± SD).

	*n*	OPG (pmol/l)	RANKL (pmol/l)
Sham	20	0.55 ± 0.05^∗^	0.53 ± 0.07^∗^
OVX	20	0.18 ± 0.06^#^	0.79 ± 0.1
OVX+ole	20	0.45 ± 0.05^∗^^,#^	0.43 ± 0.13^∗^^,*Δ*^
OVX+E2	20	0.47 ± 0.04^∗^^,#^	0.55 ± 0.11^∗^

^∗^ *P* < 0.05 vs. OVX group; ^#^*P* < 0.05 vs. sham group; *^Δ^P* < 0.05 vs. OVX+E2 group.

## Data Availability

The datasets used and analyzed during the current study are available from the corresponding author upon reasonable request.
